# Appointment Scheduling Problem in Complexity Systems of the Healthcare Services: A Comprehensive Review

**DOI:** 10.1155/2022/5819813

**Published:** 2022-03-03

**Authors:** Ali Ala, Feng Chen

**Affiliations:** ^1^Department of Industrial Engineering & Management, Shanghai Jiao Tong University, Shanghai, China; ^2^Sino-US Global Logistics Institute, Shanghai Jiao Tong University, Shanghai 200240, China

## Abstract

This paper provides a comprehensive review of Appointment Scheduling (AS) in healthcare service while we propose appointment scheduling problems and various applications and solution approaches in healthcare systems. For this purpose, more than 150 scientific papers are critically reviewed. The literature and the articles are categorized based on several problem specifications, i.e., the flow of patients, patient preferences, and random arrival time and service. Several methods have been proposed to shorten the patient waiting time resulting in the shortest idle times in healthcare centers. Among existing modeling such as simulation models, mathematical optimization techniques, Markov chain, and artificial intelligence are the most practical approaches to optimizing or improving patient satisfaction in healthcare centers. In this study, various criteria are selected for structuring the recent literature dealing with outpatient scheduling problems at the strategic, tactical, or operational levels. Based on the review papers, some new overviews, problem settings, and hybrid modeling approaches are highlighted.

## 1. Introduction

Today, it is widely recognized that a well-designed healthcare process must provide timely and easy access to healthcare facilities for all patients [1]. Appointment Scheduling (AS) can enhance the utilization of expensive staff and facilities' medical resources while reducing patient wait times. Appointment scheduling aims to build an appointment system that optimizes a specific quality standard in a healthcare application of scheduling tasks under uncertainty. The primary function of healthcare management programs is to minimize patient waiting times in public hospitals and increase patient satisfaction [2]. Healthcare services coping with a large number of outpatients may have several obstacles to address. For instance, a long waiting period for a treatment negatively impacts the patient's experience and may diminish the quality of care [3]. In general, healthcare centers such as hospitals and clinics accumulate an increasing number of patients needing their services. Hospitals have to implement quick and effective healthcare facilities to accommodate new patients and keep people patronizing them [4]. They must successfully identify the bottlenecks, anticipate the effect of diversity on-demand, and compute the optimal capacity distribution [5]. Healthcare centers are evaluated by recognizing the best methods, applying measurable techniques, and having an obligation to improve. Healthcare clinics use decision support systems to provide low-cost and assessable services to individuals to preserve the care quality of services [6]. The solutions presented in the literature aim to reduce waiting times by developing decision support systems to manage outpatient clinic services [7]. Over recent years, healthcare systems have been strained to provide patients with high-quality services despite insufficient funding. One of healthcare's most important issues, ASP, has improved quality and prompt access to health facilities. Time is an essential element in ensuring patient safety and performance, and time is a crucial determinant of patients' satisfaction [8].

In principle, the purposes of ASPs can be divided into four categories: decreasing service costs, increasing patient satisfaction, reducing waiting time, improving fairness, and reducing costs in healthcare [9]. One of the central issues in healthcare is fairness, which is a primary concern when scheduling patients and doctors [10]. Aside from fairness in scheduling, further encouragement is attained through a novel gain framework unique to the division and was not reported previously. Another critical issue on fairness is mending personal scheduling preferences [11]. The appointment scheduling's main problem is optimizing healthcare resources by improving human resources and medical equipment utilization, leading to the depreciation of the patient waiting times. Several studies have shown that the primary explanation for patient dissatisfaction in outpatient scheduling is often extended waiting time, and fair waiting times are required based on clinical competence [12]. Simulation models are among the most well-known approaches to investigating random factors' influence on patients' waiting time and doctors' idle time in appointment scheduling [13]. The optimization model uses a Simulated Annealing method to optimize the patient appointment scheduling mitigating the average service period and whole patient waiting times. According to the obtained result, the entire service time and the patient waiting time have been reduced by about 5% and 38% compared with the current situation, respectively [14, 15]. They examined the quality of their solutions via structural results and compared them with heuristic scheduling practices using a discrete event simulation. Some scholars [16, 17] applied for advanced work inside the literature to layout models to maximize the variety of patient appointments, minimize affected patient waiting time, and increase patient satisfaction. They also defined the answer set programming to solve the proposed combinatorial optimization problem that exhibited a suitable assessment used in artificial intelligence [18–20]. This paper provides an overview of the no-show problem from the following perspectives: Our contribution in this review study is to assess and examine all scientific work in appointment scheduling from 2000 to 2021, emphasizing complexity techniques. In investigating patient admission scheduling with varied applications, we examine several types of problem descriptions.

Furthermore, we also review the works available in solving other healthcare scheduling, including waiting time, using artificial intelligence, and queuing theory in appointment scheduling. Our review work centered around appointment scheduling in the complexity of healthcare research considering this problem is the most studied healthcare scheduling problem as described, concentrating on various methods used in ASP to decrease waiting time and improve patient satisfaction in healthcare. The remainder of this paper is organized as follows.

Section 2 reviews the existing articles on outpatient scheduling problems and related works.  Section 3 presents the broad performance criteria of the present methodologies in appointment scheduling problems.  Section 4 discusses various application domains and healthcare application methods, while the patients' choice function has more areas. An affected person chooses a selected provider (which determines carrier fine and health facility revenue), a specific day of the week (carrier delay), and a particular time of appointment (convenience). Finally, the findings and conclusions for future guidance are discussed in Section 5.

## 2. Research Methodology

This search aims to uncover papers that seek to determine patients who will turn up for their appointments. As a result, the search is initially limited to articles focusing on the keyword emergency or its synonyms. The comprehensive review is based on the publications related to the issue of appointment scheduling published from 2000 to 2021 in the Web of Science (*WoS*) Core Collection database. As can be seen, the number of recent articles has overgrown.  Figure 1 shows the percentage of application domains to the patient and outpatient scheduling problems. As can be seen, most of the existing outpatient appointment scheduling applications are in the field of chemotherapy and radiotherapy. Hence, we recommend a pie chart about different healthcare branches handling the green outpatient scheduling inside a radiotherapy department defined in such a manner to represent different actual-existence situations. The effectiveness of discussed studies is evaluated on randomly generated issues and a real case situation. The outcomes are very encouraging since the developed optimization models can overcome human experts' performance.

As seen in Figure 1, appointment scheduling has been discussed in many literature review topics. Generally, the problems are based on highly aggregated information at various times of the year. Nearly half of the contributions are seen in or after 2013, illustrating the increasing topics for researchers in the appointment scheduling program. Since the total number of manuscripts is massive, we restrict manuscripts to those posted in or after 2014 and 2015. The number of papers published in English regarding this issue between 2014 and 2015 is limited. However, the number of articles published after 2015 has risen due to the contribution achieved between researchers and the healthcare sector. They realized that they could benefit from this system's advantages, including better working time for staff and suitable follow-up for ordinary patients with chronic illnesses.

In Figure 2, we have also considered different publication indexes in appointment scheduling, such as SCI (blue), SJR (orange), IOS (grey), and JCR (yellow). As we can see, the number of papers from 2000–2021 on the SCI and JCR has increased slightly, and it has shown that many authors are believed to publish the article in some well-reputed journals. However, the Appointment scheduling topic is also going viral for many scholars these years as it is essential for healthcare services and management.

Also, in Figure 3, author keywords were more likely to define the difficulties and methods. In contrast, keywords plus included general terms like “appointment Systems,” “health care,” “arrival time,” “WTS,” and pleased. *VOSviewer* is used to display the cooccurrence connection of the network of the 200 keywords. The node's scale indicates the frequency of the keywords, and the thickness of the line indicates the vicinity of the relationship between the three main keywords. Three frequently used terms, “Appointment scheduling,” “optimization,” and “Healthcare,” are highlighted in the center with a more prominent label and a circle. In the graphic, the difference between the two keywords reflects the similarity of the words in terms of the connections. For instance, the keyword “Healthcare” appeared with numerous other terms such as “Systems,” “Optimization,” “admission,” and “arrival time.” As a result, the keyword placement is determined by the number of other keywords that share positive similarities. The cooccurrence map reveals that simulation in appointment scheduling comprises a broad spectrum of issues, including the emergency department, hospital planning network, operation, outpatient capacity planning, appointment scheduling, and resource allocation. The smaller nodes, which are associated with keywords such as “time delivery,” “algorithm,” “fairness,” “discharge,” “delays,” and “performance,” represent the lower cofrequency of these words across the examined papers, despite their tight connection with the Appointment scheduling.

It also depicts the current patients' scheduling core elements in operation research (OR). The number of articles in which the keywords appear to be together, recreating the connection of their different research areas, is used to calculate the strength of the link between two keywords. This contribution has made it possible for researchers in this area to pick up more novel and appealing topics.  Table 1 presents a list of outpatient scheduling models and methods' taxonomy. Most of the literature addresses modeling approaches presented earlier in this review paper that considered obtaining stability between patients' wait time and doctors' utilization through a hospital consultation and resources. In reality, direct and indirect waiting time is one of the initial practical factors in appointment scheduling. However, this modeling is difficult for the whole process for many reasons. First, unlike the direct waiting period during which the appointment is stopped is a typical ending; waiting time issues are more realistically modeled as unlimited problems. Second, outpatients are assigned an appropriate appointment time to select several preferred providers in a scheduling problem. Also, ASPs made for a specific doctor are coupled with different days and doctors on an actual day.

## 3. Results and Analysis

There are many techniques in the healthcare research areas. One of the crucial areas is utilizing appointment scheduling. In this section, some methods are analyzed to determine which method is more efficient than the others with their advantages as bases. The admission process is introduced with or without appointment only by the online or call services. The fundamental goal is to minimize access time by assigning part of the resources to patients who call for scheduling on the same day or within a few days [31, 32].

### 3.1. Overlapping Scheduling (OLAS)

The overlapping appointment scheduling (OLAS) model shortens the patient waiting time and the doctor's idle time in an outpatient healthcare hospital with a stochastic service time while maximizing the doctor's utilization and patient satisfaction [33–35]. OLAS model refers to deciding the optimal overlapping periods between the patient appointment and allocated service times. OLAS is usually formulated as an optimization problem to minimize the total cost of patients waiting and doctors' idle time, given the probabilistic distributions for patient flow and the service time [36, 37]. This discovery should help improve clinic services and ensure service quality [38]. Another study at the University Hospital of Egypt [39] analyzed patients' satisfaction with the quality of services in outpatient clinics, concluding that there is a need for continuous quality improvement and care in the healthcare environment, mainly to satisfy patients. The process of developing an overlap period in clinics with different assumptions is related to the service time distribution, over time, and no-shows [40, 41]. OLAS's primary advantages for appointment scheduling are its lack of specific scheduling services, such as alarm and warning of overlapping times. In general, OLAS increases productivity and profit despite the expense of additional staff. Also, some appointment analyses emphasize the importance of the number of operation researches. The OLAS model's objective is to determine the effect of overlapping appointments in a healthcare sector (clinic) setting. Different units are involved in this process [42, 43].

### 3.2. Markovian Scheduling Method (MSM)

The queueing theory has numerous applications in the field of healthcare management. Because they play such a significant role in hospitals, the research of queuing systems has often focused on the busy period and waiting time. A queuing system is typically defined as a patient entering a queue, being served at a service point by a server (doctor), and then exiting the row [44]. A stochastic process, a type of embedded Markov chain, governs the state-to-state transitions. At the same time, a different probabilistic mechanism determines the time spent in each stage. The transition probabilities are assumed to depend on the current state, and the time spent in each step is considered to depend on the present and following conditions [45, 46]. Many researchers use Markovian methods to investigate service scheduling research, such as for ambulance unloading delays, a Markovian queueing model was used [47, 48]. Another analysis that used the Markovian model to estimate patient services was the basic Markovian model's waiting time in a hospital using order statistics [49, 50]. The Markovian models show that a healthcare condition often depends on the standard sequence of carefully followed steps. These actions can formulate the difficulty, purpose of study, data gathering, concept and validation, and the network model's systems. Markovian chain method for appointment scheduling has conceived a new idea wherein knowledge about that approach depends on one or two booking agents' expertise [12]. The Markov decision model's different number of sessions and duration determines an optimal policy for a given problem. For instance, the number of semiurgent patients scheduled in a particular week, given the expected demand or the number of appointment scheduling patients, considers walk-in patients' anticipated direction [51, 52]. In both cases, it is assumed that the number of this week's patient arrivals is not influenced by the number of patients who arrived last week. We also investigated these two healthcare methods (OLAS) and (MSM) based on how some others considered these in their work.

Based on the investigation in Table 2, we have shown that most of the papers on appointment scheduling between 2021 and 2022 are applied. Markovian systems other than OLAS as that model have many subsections to use various optimizations methods such as Mixed Linear Integer Programming (MILP), stochastic technique, and queuing theories.

The most significant difference between the Markov chain models and other approaches is patients' status during a specific period of time [60, 61], called different wait time penalties. A key factor is the order of patient treatment, i.e., first-come-first-serve (FCFS). In the case of a high number of patients requesting the care services, the ordered patients arriving later might be scheduled before those visiting earlier, thus causing the system to increase its “rate of service.” However, enforcing fairness reduces flexibility, which is called different wait time targets. The fairness policy is motivated by expediting early arrivals rather than scheduling late arrivals ahead of them [62, 63]. Furthermore, it observed that an individual's waiting times are more variable for the contemporary approach than for the sequential one; this notable feature illustrates the difference in fairness [64] (Table 3).

### 3.3. Simulation-Based Complexity of Healthcare

Simulation models are rapidly becoming a well-known approach for dealing with healthcare appointment scheduling concerns and issues. Different simulation methods were investigated in most instances. The complexity of healthcare systems arises from their complex structure, which includes the concepts of queues and flows and social systems and decision making. Modeling complex systems at the personal level rather than the population level may be more beneficial with DES as an operational research technique. Individual entities travel through a succession of discrete events one by one at discrete intervals, among which they must wait in queues because of the limited availability of resources. The simulation approaches for outpatient scheduling problems are categorized mainly in Discrete events, Agent base simulation in healthcare problems, and those are recently widely used on this topic. As reported in the pie chart in Figure 3, most articles use discrete-event simulation (DES) techniques to improve patients' services to reduce the wait time in healthcare centers. As these two methods are mainly considered in most papers, we evaluated their differences in healthcare systems. Discrete event simulation and Agent-based simulation (ABS) have capabilities and limitations. DES and ABS methods are argued to be complementary to each other. Most healthcare systems are based on two major elements; the concept of queues and flows and decision making. DES models can consider the idea of queues and flows, while ABS models can capture human behaviors and decision-making in healthcare systems. A framework for a hybrid model of DES and ABS was proposed to capture both significant elements of healthcare systems.

Also, having those simulation approaches categories for appointment scheduling, discrete-event simulation is a flexible strategy tailored to shape the methods required to notify healthcare scheduling. It allows a broad set of tools than the Markov standard method and enables the development of techniques at a depth suitable to the problem. Its dangers are few and without problems mitigated, bringing our field towards necessities for powerful modes that decision-makers can trust. Most discrete-event simulation has programmed Any Logic or Simulation Arena software to control the clock [112]. Also, adequately scheduled activities and recognizing the subsequent ones appear to allow for dynamic entities, assigning input variables, and acting technique activities appropriately.

Agent Base Simulation can also model complicated, stochastic, and nonlinear conditions and focus on specific patients. So based on the pie chart in Figure 3, we will determine these prior years; most of the simulation approaches on ASP have various percentages of each approach. On the other hand, DES varies from ABS in three different ways [113–116]: first, in the method, decision-making actions engage in ABS; second, in its depiction of queuing; and third, in the increased number of tools available to it. Patients that arrive early, late, or on time for their scheduled appointment may be addressed by the hybrid simulation model (HSM) and SO [117–120]. The most notable distinction between the HSM and SO approaches is patients' status at a certain point, referred to as differing wait time penalties. The order of patient care, i.e., FCFS, is important. [121–123]. If many patients need care services, the ordered patients who arrive later may be scheduled ahead of those who come earlier, causing the system to enhance its “rate of service.” This study proposes a combination of ABS [124–126] and nonlinear mixed-integer programming (MIP) to reduce WTS in Ass [127–129]. ABS [130] updated their concept for broad adoption, and it has been effectively implemented at ten ASs and several hospital units. The machine-learning framework integrates patient information and matching therapies, which detects trends in the simulation platform. As a result, agents offer problematic symptoms to care providers in the form of recurrent patients whose complaints were possibly mistreated in previous visits to appointment scheduling. This ASP study highlights the type of uncertainties: one about the issues involved in the activities, one about the frequency of the tasks, and one about the available resources and employs fuzzy logic to deal with these uncertainties [131, 132]. The study divides agents into two types: software and physical. The latter refers to those who can act on their initiative, including everyone from doctors and patients to healthcare workers, nurses, and other hospital personnel.

### 3.4. Queuing Theory

In theory, the typical queuing problem in appointment scheduling has long been a source of consternation for domestic and international specialists and scholars. Queue theory and accompanying better models have been frequently operated to overcome this challenge. This section adds to the theoretical optimization of queuing problems in hospital management and gives an analysis and decision-making mechanism for enhancing hospital queuing theory and medical service efficiency. The following four essential characteristics are usually used to describe the queuing system.

#### 3.4.1. Patient Arrival Mode

The time it takes for patients to show up at the queuing system is either predictable or unpredictable. The majority of patients in the hospital's queue system arrive randomly. At this moment, the arrival rule of patients entering the procedure is called admission arrival. The focus of queue theory is also on this circumstance.

#### 3.4.2. Service Model

Patient service hours are deterministic or random, and most service hours are random. The probability distribution often describes the time rule of patients receiving services.

#### 3.4.3. Queuing Rules

Healthcare for emergency patients is among the first-come, first-served services. Whenever a patient with a higher priority appears to the system, the patient getting the service must stop and be changed to treat such patients, such as the hospital emergency department for severely ill patients.

#### 3.4.4. Number of Bed Resources

A service system is typically comprised of one or more service stages. Patients' hospital diagnosis frequently necessitates many service phases, such as outpatient visits. After making an appointment, outpatients come to the queue (i.e., the waiting list, arrival time, and idle time) in a first queueing system. When the patient's appointment time arrives, they are withdrawn from the waiting list and placed into a second queueing system. The patient enters the queue at the service facility, receives the accurate service, and then departs the appointment scheduling slot in this separate queueing system. Throughout the present paper, both queueing systems will be referred to as the appointment generating queueing system and the service facility queueing system (see Figure 4).

The most widely used queuing system is the *M/M/s* or Erlang delay model for outpatient scheduling waiting time study. This model assumes a single queue with an unlimited waiting room that feeds into *s* identical servers. It is usually assumed that the patients arrive according to a Poisson process with a constant arrival rate, and the service duration follows an exponential probability distribution. The primary use of the M/M/s method includes only three variables and could be used with little internal data to produce output estimates [73, 133]. At the same time, it provided the average arrival rate, the average length of support, and several services. Also, to achieve performance measures such as the probability that arrivals will encounter a significant or average delay, a priority queueing model could be suitable if a facility intends to identify the ability required to assure a centered service level for the best precedence customers [134]. For example, Queuing analysis is also an essential method in predicting ability needs for potential future situations, including demand rises due to emerging or urgent new illnesses, wanting a physician's care more quickly to prevent extreme scientific consequences [135, 136].

### 3.5. Artificial Intelligence (AI)

Healthcare is one of the research sectors in which Artificial Intelligence (AI) has high potential advantages. Recently, more state-of-the-art AI methods has been addressed through appointment scheduling. In order to improve the efficacy of scientific operations, numerous solutions have been introduced for online systems, appointment/surgical procedure scheduling, medical image analysis, and treatment plan and forecasting of uncommon diseases, and AI is easily carried out in appointment scheduling. The software can significantly affect the ultimate use of resources by considering these various demanding situations in a hospital's everyday working surroundings. AI-based scheduling Machine Learning (ML) models have a significant possible role in improving hospital healthcare services [78]. ML can maintain even more complicated models that can change several areas simultaneously, as in the postanesthesia treatment unit and surgical centers. Models of AI, which have significant economic consequences, may also restrict another organizational problem [137, 138].

Also, any bias against an underrepresented institution in an information set will result in a biased computerized decision. For example, an appointment scheduling software program can make racially discriminatory scheduling decisions. AI programs in healthcare need to avoid such inequalities. AI provides a lead to assuming the fundamentals of AI technologies (machine learning, healthcare) and their proper use in healthcare. It also offers practical support to help decision-makers promote an AI approach that can support its digital healthcare transformation. All investigation outcomes are tracked by AI, which then analyzes patterns to optimize future interactions [139, 140]. The AS system optimizes and duplicates the factors that lead to positive results. Each patient engagement is triggered by AI depending on the patient's specific needs. Using AI in the appointment scheduling system can then send out evaluations to patients via e-mail or text message, collecting feedback on the services. The system can then examine this data to identify areas where there is room for development and pass them on to the appropriate doctors. Several hospitals use AI to predict the number of patients to the emergency department two or three days in advance, allowing them to take proactive action in staffing and resource allocation [141–143]. Also, [144] examined the difficulties and prospects for hospitals to integrate AI into strategic planning and become intelligent systems with feedback-controlled operations and procedures (closed-loop systems). They [145] presented a model in healthcare scheduling during the COVID-19 outbreak healthcare service. They built on a considerable amount of theory and research on behavioral Internet of Medical Things, big healthcare data analytics, and artificial intelligence-based diagnostic algorithms, Creating a framework for categorizing artificial intelligence. For the sake of the analysis, we separate between care levels (primary, secondary, and tertiary care), planning levels (strategy, operational, and functional), and user groups (doctors, nurses, technicians, patients)

#### 3.5.1. Optimization Methods with AI

This review gives a broad overview of artificial intelligence's role in healthcare. This review does not touch on all healthcare areas that benefit from optimization modeling. However, we have suggested a range of optimization and neural networking applications to healthcare research. These optimization methods have been recently utilized in many optimization methods. However, in healthcare, scheduling is considered more such as convolutional neural networks (CNN), recurrent neural networks (RNN), artificial neural networks (ANN), Ant Colony Optimization (ACO), Genetic Algorithm (GA), Particle Swarm Optimization (PSO), and Whale Optimization Algorithm (WOA).

Based on what we have investigated in Table 1, we have different methods of artificial intelligence, and as we can see recently, many papers have considered appointment scheduling that utilized PSO and WOA. At the same time, the rest of the areas of the neural network are primarily used in different healthcare areas.

Many scholars have investigated Particle Swarm Optimization (PSO) in their research because this method is a swarm-based intelligent stochastic search technique encouraged in different ways in healthcare scheduling. Consequently, for the versatility of numerical experimentation, PSO has been chiefly applied to address the diverse kinds of optimization problems. The PSO algorithm could be utilized to solve various healthcare scheduling issues. The first entails optimizing the problem's objective function, while the second entails optimizing the cost function of a healthcare system. In different problems, good results are achieved, confirming the PSO method's efficiency over other AI methods. As we can see in Figure 5, during 2021–2022, many papers, especially in AI and healthcare, have been collected based on PSO with a greater number of publications than other methods in such a healthcare scheduling. Also, we still have some papers from WOA and ACO that form optimization methods that stand behind the PSO methods.

Moreover, the application sets for the outpatient scheduling problem are categorized in Table 1. The implementations' scope is pervasive, varying from patient scheduling, clinical applications, and medication schedules. In the case of a clinical emergency, it is so significant, for example, for an ambulance to reach the base as fast as possible. The patient waiting time in this situation is an essential indicator of healthcare performance [144, 145]. In the case of a scientific emergency, the number of distances is critical for ambulance offerings to reach the site as quickly as possible. In this example, the patient waiting time is a crucial indicator of ambulance system performance. With the upward thrust within the cost of providing first-rate fitness care, hospital and health facility administrators practice price containment by minimizing assets for health care provisions while still striving to provide the best health care for patients. This dilemma is becoming quite prevalent within the health care network, as indicated via the massive frame of literature that analyzes the allocation of scarce health care resources. The fundamental aim is to decrease the operational cost subject to constraints, i.e., maximum vehicle size and maximum waiting time for a patient. It pointed out that the customer waiting time can be reduced by sharing the link between a set of vehicles [146].

As shown in Table 4, various review articles have collected essential appointment scheduling applications using simulation, optimization, queuing theory, and artificial intelligence methods. The desired number of keywords in each application is indicated.

## 4. Discussion

The scheduling of appointments is a complex combinatorial subject. Since the problem was initially described in its solution, it has allowed patients to be assigned to particular slots or beds in specific relevant departments. At the same time, they allow patients' demands to be addressed to the highest standards possible to ensure that all healthcare limitations are fulfilled. Patients are usually assigned to beds by a centralized admission office, which contacts departments several days ahead of time to ensure effective appointment scheduling. As mentioned in Section 3.1 to 3.5, we have focused on addressing the practices and methods to decrease or resolve appointment scheduling problems. Scholars aspire to continue further investigating the research directions in this field. Appointment scheduling can be accomplished by developing a numerical or simulation model of the booking process, optimizing service resource setup. Many academics have explored the modeling of appointment systems and scheduling algorithms with excellent results. They thoroughly examined the current state of research on associated optimization problems, optimization methods, and models in the healthcare outpatient appointment system [148, 150]. If service time follows an exponential distribution, they considered that each patient had a predetermined probability of ASP [151]. A sequential appointment plan was used to estimate the number of bookings and the scheduled service time to maximize overall service revenue. Customers' priorities are continuously variable in the service system. The literature review discussed above significantly improves the quality of outpatient facilities of the various departments studied in the healthcare clinic. The main contribution is developing a patient-oriented appointment cycle focused on multiple approaches such as scheduling, modeling, and artificial intelligence and fit to improve the efficiency of the outpatient care system. The length of care depends on the patient's characteristics and varies greatly [145]. Still, we have reviewed numerous papers and several of those models and presented the benefits; nevertheless, determining which one is more efficient is difficult. Many researchers in this field have done simulation work, and we may infer that discrete event simulation has the most benefits and a better concept of solving the constraints. In general, discrete event simulation is a very flexible approach tailored to coordinate the procedures required to implement healthcare scheduling. It also delivers a larger scale than traditional Markov chain optimization, making the model ideal for the problem. Due to different service demands and various priority levels, patient scheduling is complicated. They created [152] a paradigm that combines stochastic service times into the scheduling problem as a first step in integrating appointment scheduling and advance scheduling. Then, they added to the existing literature by presenting analytical and experimental results for the case of multiclass, multipriority patients with predictable service times.

To settle for the additional waiting time created by appointment scheduling, the provider will approve the service requirement of arrival time. They analyzed [153–155] capacity allocation and appointment scheduling in the presence of arrival time and developed a connect rule dealing with helping to address decisions. Regarding how many slots to reserve for arriving and scheduled patients, the clinic session was given a fixed daily capacity to reduce missed appointments. They developed a finite-state Markov decision model and provided the best acceptable guidelines for determining which types of arriving patients are sufficient [149, 156, 157]. The experimental results show that when the arrival intensity of outpatients does not exceed 20% of the service intensity, accepting all is the best choice. This could be an essential route for future research.

Furthermore, another important research trend is developing a forecasting model to provide new information on the interrelationships of predictors and the conditional probability of forecasting appointment scheduling using machine learning. To examine the probabilistic links between prediction factors in appointment scheduling research, Topuz [147] built the Bayesian belief network. The predictive models may be linked to the scheduling workflow, and risk assessments can be produced based on various parameters.

### 4.1. Limitations and Objectives

The study demonstrates that appointment scheduling has shifted significantly from the setting indicated by the operations-research literature. Methods based on system flexibility and variability decrease appear more feasible than quantitative optimization, particularly in high complexity and uncertainty conditions. Also, the complexities of healthcare can describe a dynamic set of operations that interact with each other. Many appointment types, times, and constraints, on the other hand, might increase total system delay because each appointment type and time generates its differential delay and queue. Eventually, minimizing complexity reduces system delays. As a result, appointment scheduling is not without constraints: Our research has certain limitations. First, a healthcare facility with a high patient waiting time enhances the fundamental scheduled gap between patients or decreases the overloading percentage. Second, in our research, the unit cost of patient waiting time, patient dissatisfaction, and physician idle time was set at values based on our consultation with the administration. On the other hand, the goal of an outpatient appointment system is to optimize existing resources, include more doctors in those departments, and reduce the length of stay time waste.

## 5. Conclusions

This study addressed existing modeling approaches for outpatient appointment scheduling in the healthcare sector. In this regard, about 150 papers are investigated better to understand outpatient appointment scheduling problems in the literature. We considered research literature from 1990 to 2020 according to the WoS database. Then the research status and development trends are summarized by bibliometrics. Based on the statistical reports generated in this study, the reader can observe the growing trend of research interest in recent years (shown in Figure 6) due to the increased hospital resources. Despite the abundant literature for outpatient appointment scheduling, there are some opportunities to improve the existing research, including developing the planning models, performance measures, and forecasting skills under different generalized conditions. For instance, more experiments can be structured to improve schedules that are carried out well on this topic. Weak schedule performance (limited performance) is because of high overbooking levels. Understanding the performance dynamics of scheduling systems could lead to developing alternative healthcare access systems. An alternative area of examination is necessary to change the status of overbooking. General public interest in improving healthcare access and service delivery will likely lead to more analysis of the existing approaches. Moreover, mathematics modeling approaches can be further used for multiple providers such as double booking, overtime costs, and to increase efficiency time among visiting doctors.

Regarding the effect of uncertain factors on outpatient waiting times, we have mentioned several practical approaches that are well-known methods in this research. Specifically, the Markovian model has difficulty in fairness policy due to the complexity of observing an individual's waiting times and a difference in various fairness factors in healthcare appointment scheduling. However, the OLAS approach is beneficial for this field because of increasing productivity obtained by overlapping time to minimize the total cost of patient waiting time and doctor idle time. It is worth mentioning that discrete-event simulation and other optimization approaches are new trends for future research. Future studies must investigate the scheduled outpatient and walk-in patient with unexpected arrival to disturb the clinic operations.

A further issue that is not often discussed openly is the discrete-event simulation approach used for accurate decision-making in healthcare. Discrete-event simulation may be mainly accurate in healthcare delivery models in place of sickness and screening applications. If a version of healthcare optimization is used, various patients need to be convinced of their benefits and limitations in the healthcare sector. Moreover, other researchers should conduct a more in-depth analysis of walk-in outpatients' effect on the punctuality of the planned arrivals. The method needs more investigation due to the complexity of this problem and could also be expanded further in terms of emergency admissions and intensive care departments. Another field of future research is to formulate the sequencing problems based on individual unpunctuality behaviors. Using a game theory approach, the extension of current models would help account for the unpunctuality between doctors, nurses, and patients. As a research gap, outpatient appointment scheduling problems could be extended to model the multistage health process, i.e., preliminary examination, drug test, and patient preparation or optimizing multiappointment schedules in clinics.

## Figures and Tables

**Figure 1:** The trend of the published articles in the area of appointment scheduling 2000–2021.

**Figure 2:** The trend of the publication based on various indexes SCI, JCR, SJR, and IOS in appointment scheduling.

**Figure 3:** The keywords for the outpatient scheduling problems.

**Figure 4:** The percentage of different simulation approaches to an outpatient scheduling problem.

**Figure 5:** Traditional queueing scheduling of appointments during the week for the patient.

**Figure 6:** Number of papers in various AI methods in appointment scheduling between 2021 and 2022.

**Table 1:** Categorizing the various artificial intelligence methods in appointment scheduling 2021–2022.

Publications	CNN	DNN	ANN	ACO	PSO	GA	WOA
Muhammad et al. [21]	*∗*						
Kumari et al. [22]						*∗*	*∗*
Shilong et al. [23]				*∗*			*∗*
Bisoy et al. [24]					*∗*		
Sarkar et al. [25]					*∗*		
Jiang et al. [26]				*∗*			
Gao et al. [27]					*∗*		
Vukobrat et al. [28]			*∗*				
Kirchohf et al. [29]	*∗*						
Nair et al. [30]		*∗*					

**Table 2:** Different methods and objectives in appointment scheduling publications between 2021 and 2022.

Publications	Markovian	Overlapping	Objectives
Ntaimo et al. [53]		*∗*	Consider stochastic programming to improve computational speed time
Mueen [54]	*∗*		Consider a fuzzy set programming and MILP to measure healthcare scheduling
Lee et al. [55]		*∗*	Practical optimization considered to solve makespan scheduling in healthcare
Zhao and Wen [56]	*∗*		Design an algorithm with a lower-bounded competitive ratio to improve patient arrival time
Xie and Liu [57]	*∗*		Continuous-time Markov chain and uniformization method to solve waiting time
Bayram and Yu [58]	*∗*		Applied Markov and newsvendor model to maximize long-run average earnings
Soodan et al. [59]	*∗*		Applied a stochastic queuing model to optimize patient arrival time

**Table 3:** The taxonomy of outpatient scheduling models and methods.

References	Mathematical optimization	Markov model	Dynamic approach	Artificial intelligence	Simulation approach	Robust approach
[65]	*∗*		*∗*			
[66]	*∗*					
[67]						*∗*
[68]	*∗*					
[69]	*∗*		*∗*			*∗*
[70]			*∗*		*∗*	
[71]					*∗*	
[72]	*∗*			*∗*		
[73]	*∗*					
[74]			*∗*			*∗*
[75]	*∗*			*∗*	*∗*	
[76]						
[77]	*∗*					
[78]	*∗*		*∗*		*∗*	
[79]					*∗*	
[80]	*∗*		*∗*			
[81]		*∗*				
[82]						
[83]	*∗*			*∗*		
[84]	*∗*					
[85]						
[86]	*∗*		*∗*			*∗*
[87]					*∗*	
[88]				*∗*		
[76]			*∗*			
[78]	*∗*					
[89]			*∗*			
[90]			*∗*			
[91]						
[92]	*∗*					
[83]						
[93]				*∗*		
[94]	*∗*					
[95]						*∗*
[96]	*∗*					
[97]					*∗*	
[98]						
[99]			*∗*			
[100]				*∗*		
[101]						
[102]	*∗*		*∗*			
[103]				*∗*		
[104]	*∗*					
[44]	*∗*					
[105]			*∗*		*∗*	
[106]			*∗*			
[107]	*∗*	*∗*				*∗*
[108]						
[109]				*∗*		
[110]	*∗*		*∗*			
[111]		*∗*				

**Table 4:** Categorizing the application domains for the outpatient scheduling models.

Application domain	Articles
Chemotherapy	[68, 73, 75, 78, 86, 87, 92, 95–99, 102, 103, 106–109, 118]
Oncology	[67, 69–71]
Radiotherapy	[66, 67, 72, 74, 76, 78, 83, 87–91, 93, 94, 101, 147]
Physiotherapy	[83–85]
Rehabilitation therapy	[77, 86, 104, 105, 111]
Hemodialysis	[79, 82, 148, 149]
Pathology	[80, 102, 110]

## Data Availability

The datasets used and/or analyzed during the current study are available from the corresponding author on reasonable request.
